# Logistic Regression Analysis of Risk Factors and Improvement of Clinical Treatment of Traumatic Arthritis after Total Hip Arthroplasty (THA) in the Treatment of Acetabular Fractures

**DOI:** 10.1155/2022/7891007

**Published:** 2022-05-04

**Authors:** Zijun Zhao, Long Feng

**Affiliations:** ^1^Department of Orthopedics, Beijing Hospital of Traditional Chinese Medicine of Huairou Hospital, Beijing, China 101400; ^2^Department of Anesthesiology, PLA General Hospital of Hainan Hospital, Sanya 572000, China

## Abstract

**Objective:**

Logistic regression was adopted to analyze the risk factors of traumatic arthritis after total hip arthroplasty (THA) in the treatment of acetabular fractures, and the clinical treatment was enhanced.

**Methods:**

A total of 200 patients with acetabular fractures treated in our hospital from February 2019 to April 2021 were enrolled for THA. According to the occurrence of traumatic arthritis after operation, the patients were divided into control group and study group. The control group was patients without traumatic arthritis (*n* = 165), and the study group was patients with traumatic arthritis after operation (*n* = 35). The general data were analyzed, the risk factors of traumatic arthritis after THA for acetabular fractures were analyzed by logistic regression, and the clinical treatment methods were promoted.

**Results:**

First of all, there exhibited no significant difference in the general data such as sex, age, medical history, and operation site (*P* > 0.05). There were significant differences in the general data of whether the patients had a job, rehabilitation exercise, and osteoarthritis before operation (*P* < 0.05). Secondly, we compared the curative effects between two groups. The effective rate in the study group was higher compared to the control group (*P* < 0.05). After treatment, the Harris hip function score of the study group at discharge, 1 month, 3 months, and 6 months after discharge was higher compared to that of the control group (*P* < 0.05). The incidence of postoperative complications in the study group was significantly higher compared to that in the control group (*P* < 0.05). The presence of osteoarthritis, curative effect, poor reduction of fracture, injury of articular cartilage, entry of internal fixation into the joint, avascular necrosis of the femoral head, and infection before operation were significantly correlated with traumatic arthritis after THA in the treatment of acetabular fractures (*P* < 0.05). Logistic regression analysis indicated that poor reduction, curative effect, articular cartilage injury, entry of internal fixation into the joint, avascular necrosis of the femoral head, infection, and preoperative osteoarthritis were the risk factors of traumatic arthritis after THA in the treatment of acetabular fractures (*P* < 0.05).

**Conclusion:**

Poor fracture reduction, curative effect, articular cartilage injury, internal fixation into the joint, avascular necrosis of the femoral head, infection, and the presence of osteoarthritis before operation are the risk factors of traumatic arthritis after THA in the treatment of acetabular fractures. When performing THA for patients with acetabular fracture, attention should be paid to the presence of osteoarthritis before operation, and for those with poor curative effect, attention should be paid to the occurrence of poor fracture reduction, articular cartilage injury, internal fixation into the joint, avascular necrosis of the femoral head, and combined infection, and timely intervention measures should be taken to reduce the risk of traumatic arthritis after operation.

## 1. Introduction

Acetabular fractures are often caused by high-energy injuries [1]. In the past, due to the relatively low incidence and lack of understanding of acetabular fractures, the treatment effect is poor. With the development of China's economy and the increase of traffic accidents, there are more patients with acetabular fracture [2]. The current point of view is that as an intra-articular fracture, the treatment principle of acetabular fracture is early anatomical reduction, effective internal fixation, and early functional exercise [1, 2]. Open reduction and internal fixation have become the gold standard for the treatment of displaced acetabular fractures [2]. Because of its complex anatomy and often associated with other site injuries, the treatment of such patients needs to be highly specialized. Even with experienced orthopedic surgeons, there are still a considerable number of patients with postoperative complications. Common complications include traumatic arthritis and osteonecrosis of the femoral head [3]. When patients have severe hip pain and limited function, surgical intervention is often needed because hip arthrodesis will lead to a series of problems, such as the loss of hip joint function and the change of spinal force; it has rarely been adopted, and joint replacement is advocated.

Total hip arthroplasty (THA) is mainly employed for late surgical treatment of patients with hip disease; its main purpose is to relieve hip pain and enhance hip function [4]. After decades of development, the materials of hip prosthesis have developed from stainless steel to cobalt-chromium-molybdenum and other alloys. With the improvement of medical level and the progress of material science, hip replacement has achieved good long-term results and gradually began to be adopted in young patients. The application in patients with acetabular fracture has also achieved good results, but there are many related complications in further follow-up, such as high revision rate, severe heterotopic ossification, and infection [5]. Traumatic arthritis is the most common complication after acetabular fracture. Through the analysis of 569 patients with acetabular fractures, some scholars reported that the overall incidence of postoperative traumatic arthritis was 17%, of which the incidence of complete reduction was 10% and that of incomplete reduction was 35% [6]. Many literatures have pointed out that the postoperative effect is not satisfactory, which is often accompanied by joint dislocation, marginal compression, and ipsilateral femoral head fracture such as in the initial operation, which failed to fix the fracture, the necessary bone graft treatment, and often bring about serious complications [7]. Based on this, this study analyzed the risk factors of traumatic arthritis after THA in the treatment of acetabular fractures by logistic regression and promoted the clinical treatment methods to provide theoretical basis for clinical treatment.

## 2. Patients and Methods

### 2.1. General Information

A total of 200 patients with acetabular fractures treated in our hospital from February 2019 to April 2021 were enrolled for THA. According to the occurrence of traumatic arthritis after operation, the patients were divided into control group and study group. The control group was patients without traumatic arthritis (*n* = 165), and the study group was patients with traumatic arthritis after operation (*n* = 35). This study was permitted by the Medical Ethics Association of our hospital, and all patients noticed informed consent. All patients were unilateral hip joint lesions, excluding preoperative severe heart, lung, and brain diseases affecting normal life, lower limb severe vascular occlusion, and knee or ankle arthritis under the influence of walking.

### 2.2. Treatment Methods

#### 2.2.1. Preoperative Treatment

Routine examination of erythrocyte sedimentation rate (ESR), C-reactive protein (CRP), X-ray of the pelvis and hip, and CT were carried out before operation, and MRI was carried out if necessary. The type of fracture, fracture healing, infection, bone defect, heterotopic ossification, osteonecrosis of the femoral head, and vascular and nerve injury were evaluated. To understand the bone mass of the affected hip, the length and diameter of the femoral head and neck, measure the length of both lower limbs. For medical diseases complicated with cardio-cerebrovascular, respiratory system, diabetes, and other medical diseases, please consult the relevant departments for treatment. There was prophylactic treatment with antibiotics and routine blood preparation the day before operation.

#### 2.2.2. Operation Method

The operation was carried out under general anesthesia. All patients in this group were treated with posterolateral approach and lateral recumbent position. In the treatment of THA, a new generation of metal-to-metal surface hip prosthesis is enrolled. The acetabular side was fixed with pearl micropore, and the femur side was fixed with bone cement. Of note, the type of femoral head prosthesis and the corresponding acetabular prosthesis were determined according to the diameter of the femoral neck. The acetabular side was pressed to fix the prosthesis at the position of anteversion 15°~20° and abduction 40°~45°. For the patients with defects, autogenous femoral head particles were given. On the femoral side, with the assistance of the central positioning guide, a guide needle was inserted along the center of the femoral head and neck, a tube file was installed along the positioning needle, the femoral head was ground and stopped at the junction of the head and neck, and the excess bone was removed with a bone knife or rongeur. After drilling on the femoral head, modulate the bone cement, place it on the surface of the femoral head and the surface of the prosthesis, and continue to press until the bone cement is solidified. After the joint replacement, the hip joint was reduced, the stability of the joint and the length of the lower limbs were checked, the intraoperative fluoroscopy was confirmed, the wound was washed, the drainage tube was placed, and the wound was sutured layer by layer.

#### 2.2.3. Postoperative Treatment

After the operation, the affected limb “D” shoes were immobilized and the mild abduction position was maintained. The incision was placed with negative pressure drainage for 48 hours, and antibiotics and anticoagulants were routinely adopted to prevent infection and deep venous thrombosis of lower extremities. Functional exercise and weight-bearing time were determined according to the type of prosthesis, bone condition, fracture healing, and bone grafting. Generally, the quadriceps isometric contraction exercise and joint passive exercise were carried out on the bed 24 hours after operation. The affected limb was loaded gradually after 4-6 weeks, and the full weight-bearing exercise began 3 months later.

### 2.3. Observation Index

#### 2.3.1. General Information

Statistics were made on the sex, age, job, medical history, rehabilitation exercise, surgical site, and preoperative osteoarthritis between the two groups.

#### 2.3.2. Curative Effect Evaluation

Effective: (1) the reduction of the fracture site is good, (2) the healing speed is fast, and (3) there are no serious complications after operation. Ineffective: (1) the reduction of the fracture site is poor, (2) the healing speed is slow, and (3) serious complications occur after operation. Effective rate = markedly effective rate + effective rate.

#### 2.3.3. Harris Hip Joint Function Score

Harris hip joint function score scale: adopted to evaluate the therapeutic effect of hip joint disease, evaluated by medical staff, including pain, function, deformity, and range of motion 4 dimensions, a total of 10 items, a total score of 100. The higher the score, the better the hip joint function.

#### 2.3.4. Incidence of Postoperative Complications

The incidence of postoperative complications was calculated between the two groups.

### 2.4. Statistical Analysis

The data of this study were analyzed by SPSS 26.0, the counting data were presented by [*n* (%)], the chi-square partition method was employed for the pairwise comparison, and the metrological data of normal distribution were presented as $\left(\bar{x}\pm s\right)$. The independent sample *t*-test was adopted for the comparison, the one-way analysis of variance (ANOVA) was employed for the comparison, and the SNK-q test was adopted for further pairwise comparison. The measurement data of skewness distribution were presented by median (minimum to maximum), nonparametric test was employed, rank sum test was adopted for rank data, repeated measurement variance analysis was employed for comparison of repeated measurement data, Person correlation analysis was adopted for normal distribution data correlation, and Spearman correlation analysis was employed for skewness distribution data and grade data correlation. Logistic regression analysis was employed to analyze the risk factors affecting the rehabilitation of motor and cognitive function in patients with stroke. *P* < 0.05 indicated that the difference had statistical significance, and *P* value less than 0.01 was viewed as highly statistically significant.

## 3. Results

### 3.1. Comparison of General Data

First of all, we compared the general data, and there exhibited no significant difference in sex, age, medical history, and operation site (*P* > 0.05). There were significant differences in the general data of whether the patients had a job, rehabilitation exercise, and osteoarthritis before operation between the two groups (*P* < 0.01). All the data results are indicated in Table 1 and Figure 1.

### 3.2. Comparison of Curative Effect Evaluation

Secondly, we compared the curative effects. The study group was significantly effective in 5 cases, effective in 18 cases, ineffective in 12 cases, and the effective rate was 65.71%; the control group was markedly effective in 105 cases, effective in 49 cases, ineffective in 11 cases, and the effective rate was 93.33%. The effective rate in the study group was higher compared to that in the control group (*P* < 0.01). All the data results are indicated in Table 2.

### 3.3. Harris Comparison of Hip Joint Function Score

Then, we compared the Harris hip function score. Before treatment, there was no significant difference, and the difference exhibited not statistically significant (*P* > 0.05). After treatment, the Harris hip function score of the study group at discharge, 1 month, 3 months, and 6 months after discharge was higher compared to that of the control group (*P* < 0.01). All the data results are indicated in Table 3.

### 3.4. Incidence of Postoperative Complications

Next, we compared the incidence of postoperative complications. The incidence of postoperative complications such as poor fracture reduction, articular cartilage injury, internal fixation into the joint, avascular necrosis of the femoral head, and infection in the study group was higher compared to that in the control group (*P* < 0.05). All the data results are indicated in Table 4.

### 3.5. Analysis of the Relationship between Postoperative Complications and Traumatic Arthritis after THA in the Treatment of Acetabular Fractures

And then we analyzed the correlation between postoperative complications and traumatic arthritis after THA for acetabular fractures. Person correlation analysis indicated that there was no significant correlation between work, rehabilitation exercise, hip function, and traumatic arthritis after THA (*P* > 0.05). The presence of osteoarthritis, curative effect, poor reduction of fracture, injury of articular cartilage, entry of internal fixation into the joint, avascular necrosis of the femoral head, and infection before operation was significantly correlated with traumatic arthritis after THA in the treatment of acetabular fractures (*P* < 0.05). The results of all the data are indicated in Table 5.

### 3.6. Logistic Regression Analysis of Risk Factors of Traumatic Arthritis after THA in the Treatment of Acetabular Fractures

Finally, we carried out logistic regression analysis on the risk factors of traumatic arthritis after THA in the treatment of acetabular fractures. Logistic regression analysis indicated that poor reduction, curative effect, articular cartilage injury, internal fixation into the joint, avascular necrosis of the femoral head, combined infection, and preoperative osteoarthritis were related to traumatic arthritis after THA in the treatment of acetabular fractures (*P* < 0.05 or *P* < 0.01). All the data results are indicated in Table 6.

## 4. Discussion

With the increase of high energy injury, the incidence of acetabular fracture is increasing year by year [8]. Because the acetabular fracture involves the important weight-bearing joint of the lower limb and is an intra-articular fracture, anatomical reduction is of great significance to maintain the function of the hip joint [9]. According to the detailed discussion of scholars on acetabular fracture, the concept of surgical treatment has been gradually established [10]. For the surgical treatment of unstable and misaligned acetabular fractures, anatomical reduction, effective internal fixation, and early functional exercise are advocated [11]. Because acetabular fractures are mostly caused by high-energy injuries, the elderly patients are often accompanied by severe osteoporosis, irreversible damage to the articular surface after trauma, the complexity of fracture types, and the difficulties of surgical exposure, as well as significant postoperative complications and other factors; the treatment of acetabular fracture is a great challenge for orthopedic surgeons [12]. Acetabular fracture is the largest weight-bearing injury of the articular surface of the whole body, and its treatment principle is the same as other intra-articular fractures, which requires anatomical reduction, firm fixation, and early joint function exercise [13]. In the past 30 years, active early open reduction and internal fixation for displaced acetabular fractures have been recognized by most scholars [14]. Although it can effectively reconstruct the anatomical structure of the acetabulum and restore its function, there are still some postoperative complications that affect the long-term efficacy due to many factors affecting the therapeutic effect, even if it is treated by experienced specialists [15, 16]. According to the literature, it is reported that the incidence of traumatic arthritis after acetabular fracture is 20~30%, and the incidence of osteonecrosis of the femoral head is 2%~10% [17]. Other complications such as nonunion, heterotopic ossification, and other complications occur from time to time, affecting joint function [17]. Traumatic arthritis is the most common complication after acetabular fracture. Poor joint reduction is the main factor. When traumatic arthritis progresses with severe pain and dysfunction, hip arthroplasty or hip arthrodesis must be carried out. Because of hip fixation after hip fusion, it is often not acceptable to patients. At present, THA is often adopted [18, 19].

As a salvage operation, THA has been proved to be effective in the treatment of late complications of acetabular fractures through a large number of clinical studies [20]. However, the results demonstrate that there is a high long-term failure rate in the treatment of such patients in the past [21]. In 1990, some scholars reported 53 patients with acetabular fractures, 55 hips were treated with THA, and 13 patients were treated with open reduction and internal fixation and were followed up for 7.5 years [22]. Finally, 10 patients needed revision surgery [23]. In terms of conventional THA, due to scar tissue, formation of ectopic ossification, obstruction of internal fixation, and so on, the survival rate of the prosthesis is lower [24]. At present, with the improvement of the reduction technology of primary internal fixation, the improvement of prosthesis technology, the understanding of its influencing factors, and the maturity of surgical techniques, the curative effect has been enhanced [25]. Meanwhile, with the progress of technology, the types of prostheses that can be employed are increasing day by day. Metal-to-metal THA has been adopted as another option for the treatment of hip osteoarthritis and osteonecrosis of the femoral head. According to the literature, in the short- and medium-term follow-up of THA, the clinical success rate has reached 94%~100% [26]. Acetabular fractures often occur in young adults, the demand for exercise is becoming larger, and the demand for joint replacement is very high.

China began to implement femoral head replacement in the 1960s and 1970s on the basis of foreign experience [27]. After decades of continuous catch-up, great progress has been made in prosthesis materials and clinical application. With the increase of patients with high-energy injuries such as traffic accidents in China, there are more patients with acetabular fractures. When such patients have osteonecrosis of the femoral head and traumatic arthritis, joint replacement has become the first choice of treatment [27, 28]. Some scholars through 11 patients with acetabular fracture after internal fixation of THA, postoperative follow-up for an average of 3 years and 5 months, all patients' hip joint function has been improved, Harris score has been significantly enhanced, and good results were achieved [28]. According to our statistics, in the patients with acetabular fractures who underwent conservative treatment or open reduction and internal fixation, after THA, the average Harris score of hips increased from 37.1 before operation to 83.2 after the last follow-up, and the excellent and good rate was 82.4%. The range of motion of hip joint has been significantly strengthened in flexion, adduction, abduction, and rotation compared with that before operation, indicating that this kind of patients would achieve good results in THA. Some scholars believed that the main factors affecting the curative effect of THA in patients with acetabular fracture were bone defects and deformities on the acetabular side [29].

With the deeper understanding of acetabular fractures, anatomical reduction, rigid internal fixation, and early functional exercise have become the principles for the treatment of displaced acetabular fractures [30]. Surgical treatment of this kind of patients can reduce the incidence of traumatic arthritis and facilitate the overall treatment effect. However, there are still more than 20% of patients with traumatic arthritis and osteonecrosis of the femoral head after operation. Through the analysis of the data of these patients, we believe that the main reasons for the failure of treatment are as follows. (1) Incomplete fracture reduction: in particular, the blood supply of the pelvis of complex comminuted fractures and old fractures is very abundant, and the callus formed more than 3 weeks later increases the difficulty of reduction. The operation of complex comminuted fracture is difficult, and part of the free bone cannot be completely reduced, resulting in uneven articular surface. (2) Combined with dislocation of the femoral head, fracture of the femoral head or fracture of the femoral neck with dislocation of the femoral head, fracture of the femoral head, or fracture of the femoral neck will affect the blood supply of the femoral head and is prone to osteonecrosis of the femoral head. The quality of fracture reduction has an important impact on the risk of osteonecrosis of the femoral head. The reduction time of dislocation also has a certain influence. In patients with dislocation of the hip, the incidence of osteonecrosis of the femoral head within 6 hours is 5%, while that of dislocation more than 6 hours is 50%. (3) The anatomical structure of the acetabulum with internal fixation is complex, and the screw cannot be implanted directly into the hip joint during the operation, especially for the inexperienced orthopedic surgeon; it is easy to implant the screw into the joint. (4) For patients with acetabular fracture complicated with injury of femoral head and acetabular cartilage. However, the healing ability of cartilage is limited, and cartilage injury is a risk factor for acetabular fracture healing. Patients with cartilage injury in the weight-bearing area of the femoral head have a poor prognosis and are more likely to develop secondary traumatic arthritis. Patients with suspected cartilage injury should be examined by magnetic resonance imaging (MRI) of the hip joint before operation to determine whether there is cartilage injury or not. (5) Patients with acetabular fractures who take corticosteroids for a long time are often accompanied by other organ injuries, and some patients need to take hormones for a long time, which can lead to osteonecrosis of the femoral head. Studies have found that patients with open reduction and internal fixation after acetabular fractures generally occur in the early stage if osteonecrosis of the femoral head and traumatic arthritis occur, while patients with conservative treatment generally occur in the late stage. We believe that in addition to the factors caused by the trauma itself, the operation to destroy the blood supply of the femoral head is a very important reason [31].

Infection is catastrophic for orthopedic patients, and it is reported that the incidence of postoperative infection in patients with internal fixation of acetabular fractures is 5.2% [32]. The internal fixation in the patient can make the infection persist and even spread to the bony structure to cause infectious bone defect [33]. For those who have undergone surgical treatment of acetabular fractures, we should first determine whether the patient has infection before joint replacement, especially when the persistent pain of the hip joint is not relieved and the progressive aggravation of the hip joint should be carefully identified [34]. The infection indexes of these patients were examined before operation. If the relevant indexes increased, bone scanning, joint puncture for bacterial culture, and neutrophil count under high-power microscope could be carried out on the rapid frozen sections of hyperplastic granulation tissue during the operation. Whether or not to remove the internal fixation should be determined according to the specific conditions, and it may not be removed if the internal fixation does not affect the operation. In the past, the anterior and lateral X-ray films of the hip joint of patients with internal fixation were taken to determine whether the internal fixation affected the operation according to the operator's experience [35]. With the development of medicine, hip joint CT was carried out in patients with internal fixation. 3D CT reconstruction and computer surgery simulation were employed to observe whether the internal fixation affected the installation of acetabular prosthesis, which strengthened the accuracy of judgment.

In summary, poor fracture reduction, curative effect, articular cartilage injury, entry of internal fixation into the joint, avascular necrosis of the femoral head, infection, and preoperative osteoarthritis are the risk factors of traumatic arthritis after THA in the treatment of acetabular fractures. When performing THA for patients with acetabular fracture, attention should be paid to the presence of osteoarthritis before operation, and for those with poor curative effect, attention should be paid to the occurrence of poor fracture reduction, articular cartilage injury, internal fixation into the joint, avascular necrosis of the femoral head, and combined infection, and timely intervention measures should be taken to reduce the risk of traumatic arthritis after operation.

## Figures and Tables

**Figure 1:** (a) X-ray at the time of injury, transverse fracture of the right acetabulum, fracture of the posterior wall of the left acetabulum, subluxation of the left hip joint, and fracture of the left pubic branch. Figure X-ray after B ORIF, bilateral acetabular fractures and pubic branch fractures were fixed with plates and screws. (b, c) X-ray, CT, dislocation of left hip joint, acetabular bone defect, articular surface collapse, formation of periacetabular osteophyte and heterotopic ossification 3 months after ORIF. (d) During the operation, the posterolateral incision indicated the defect of the posterolateral wall of the left acetabulum and bone resorption. Structural bone graft and screw fixation of bone graft. (e) During the operation, the acetabulum was fixed with titanium mesh and screws. (f) During the operation, the bone cement was filled, the liner was placed, and the biological stalk was implanted on the side of the femur. (g) C-arm perspective during the operation, the position of the prosthesis is acceptable and the angle is normal. (h) X-ray examination was carried out after operation. (i) Recent follow-up X-ray indicated that there was no loosening, displacement, and wear of the prosthesis.

**Table 1:** Comparison of general data between two groups of patients [*n*/%].

Group	C group (*n* = 165)	R group (*n* = 35)	*χ* ^2^	*P*
Gender				
Male	82 (49.70)	18 (51.43)	0.034	>0.05
Female	83 (50.30)	17 (48.57)		
Age				
<30	25 (15.15)	7 (20.00)	0.809	>0.05
30-60	107 (64.85)	20 (57.14)		
>60	33 (20.00)	8 (22.86)		
Work				
Yes	102 (61.82)	14 (40.00)	5.642	<0.01
None	63 (38.18)	21 (60.00)		
Medical history				
High blood pressure	16 (9.70)	2 (5.71)	1.079	>0.05
Diabetes	13 (7.88)	4 (11.43)		
Hyperlipidemia	18 (10.91)	3 (8.57)		
Rehabilitation exercise				
Yes	148 (89.70)	12 (34.29)	55.411	<0.01
No	17 (10.30)	23 (65.71)		
Operation site				
Left side	79 (47.88)	19 (54.29)	0.474	>0.05
Right side	86 (52.12)	16 (45.71)		
There is osteoarthritis before operation				
Yes	20 (12.12)	31 (88.57)	88.834	<0.01
No	145 (87.88)	4 (11.43)		

**Table 2:** Comparison of curative effect between two groups of patients [*n*/%].

Group	*N*	Significant effect	Effective	Invalid	Efficiency
C group	165	105 (63.63)	49 (29.70)	11 (6.67)	154 (93.33)
R group	35	5 (14.28)	18 (51.43)	12 (34.29)	23 (65.71)
*χ* ^2^					21.642
*P*					<0.01

**Table 3:** Comparison of Harris hip joint function score between the two groups $\left[\bar{x}\pm s,\text{points}\right]$.

Group	*N*	Before treatment	When discharged from the hospital	One month after discharge	3 months after discharge	6 months after discharge
C group	165	56.66 ± 4.31	65.32 ± 3.44	78.72 ± 2.66	86.65 ± 3.31	90.77 ± 3.21
R group	35	56.22 ± 4.64	60.53 ± 3.56	68.93 ± 4.12	75.21 ± 3.64	80.23 ± 3.43
*t*		0.541	7.437	17.758	18.246	17.433
*P*		>0.05	<0.01	<0.01	<0.01	<0.01

**Table 4:** Comparison of the incidence of postoperative complications between the two groups [*n*/%].

Group	*N*	Poor reduction of fracture	Articular cartilage injury	Internal fixation enters the joint	Avascular necrosis of femoral head	Combined infection	Total incidence rate
C group	165	1 (0.61)	1 (0.61)	1 (0.61)	1 (0.61)	1 (0.61)	5 (3.05)
R group	35	3 (8.57)	5 (14.28)	3 (8.57)	4 (11.44)	5 (14.28)	20 (57.14)
*χ* ^2^							77.303
*P*							<0.05

**Table 5:** Analysis of the relationship between postoperative complications and traumatic arthritis after THA in the treatment of acetabular fractures.

Factors	*r*	*P*
Work	0.154	>0.05
Rehabilitation exercise	0.235	>0.05
There is osteoarthritis before operation	0.584	<0.05
Curative effect	0.783	<0.05
Hip joint function	0.165	>0.05
Poor reduction of fracture	0.842	<0.05
Articular cartilage injury	0.783	<0.05
Internal fixation enters the joint	0.695	<0.05
Avascular necrosis of femoral head	0.842	<0.05
Combined infection	0.886	<0.05

**Table 6:** Logistic regression analysis of risk factors of traumatic arthritis after THA in the treatment of acetabular fractures.

Factors	*b*	SE	Chi-square value	*P*	OR	95% CI for OR
There is osteoarthritis before operation	2.452	0.678	13.079	<0.01	11.612	3.074-43.855
Curative effect	2.151	0.982	4.798	0.028	8.593	1.254-58.893
Poor reduction of fracture	2.894	1.021	8.034	0.005	18.065	2.442-133.641
Articular cartilage injury	0.566	0.122	21.524	<0.01	1.761	1.387-2.237
Internal fixation enters the joint	0.982	0.125	61.717	<0.01	2.670	2.090-3.411
Avascular necrosis of femoral head	0.583	0.053	121.000	<0.01	1.791	1.615-1.988
Combined infection	1.563	0.356	19.276	<0.01	4.773	2.376-9.590

## Data Availability

No data were used to support this study.
